# Thermoase-Derived Flaxseed Protein Hydrolysates and Membrane Ultrafiltration Peptide Fractions Have Systolic Blood Pressure-Lowering Effects in Spontaneously Hypertensive Rats

**DOI:** 10.3390/ijms151018131

**Published:** 2014-10-09

**Authors:** Ifeanyi D. Nwachukwu, Abraham T. Girgih, Sunday A. Malomo, John O. Onuh, Rotimi E. Aluko

**Affiliations:** 1 Department of Human Nutritional Sciences, University of Manitoba, Winnipeg, MB R3T 2N2, Canada; E-Mails: nwachuki@myumanitoba.ca (I.D.N.); malomos@myumanitoba.ca (S.A.M.); onuhj@myumanitoba.ca (J.O.O.); 2 Richardson Centre for Functional Foods and Nutraceuticals, University of Manitoba, Winnipeg, MB R3T 2N2, Canada; E-Mail: umgirgia@myumanitoba.ca

**Keywords:** antihypertensive, hypertension, bioactive peptides, thermoase, flaxseed, angiotensin converting enzyme, renin, spontaneously hypertensive rat, membrane ultrafiltration, systolic blood pressure

## Abstract

Thermoase-digested flaxseed protein hydrolysate (FPH) samples and ultrafiltration membrane-separated peptide fractions were initially evaluated for *in vitro* inhibition of angiotensin I-converting enzyme (ACE) and renin activities. The two most active FPH samples and their corresponding peptide fractions were subsequently tested for *in vivo* antihypertensive activity in spontaneously hypertensive rats (SHR). The FPH produced with 3% thermoase digestion showed the highest ACE- and renin-inhibitory activities. Whereas membrane ultrafiltration resulted in significant (*p* < 0.05) increases in ACE inhibition by the <1 and 1–3 kDa peptides, only a marginal improvement in renin-inhibitory activity was observed for virtually all the samples after membrane ultrafiltration. The FPH samples and membrane fractions were also effective in lowering systolic blood pressure (SBP) in SHR with the largest effect occurring after oral administration (200 mg/kg body weight) of the 1–3 kDa peptide fraction of the 2.5% FPH and the 3–5 kDa fraction of the 3% FPH. Such potent SBP-lowering capacity indicates the potential of flaxseed protein-derived bioactive peptides as ingredients for the formulation of antihypertensive functional foods and nutraceuticals.

## 1. Introduction

Hypertension is not only a major risk factor for cardiac, cerebrovascular and other vascular diseases [1], it is also considered a leading cause of mortality worldwide with over 7 million deaths and 92 million disability-adjusted life years recorded annually [2]. The renin-angiotensin-aldosterone system (RAAS), which is an important signaling pathway credited with the regulation of extracellular fluid volume, arterial pressure, and tissue perfusion has received significant attention from investigators recently because of its potential as an excellent target for blood pressure lowering agents [3,4,5,6]. Renin and angiotensin I-converting enzyme (ACE) play key roles in the RAAS pathway; renin is responsible for catalyzing hydrolytic production of the inactive decapeptide angiotensin I (AT-I) from the *N*-terminus of the plasma protein angiotensinogen in what has been recognized as the initial and rate-determining reaction. ACE subsequently cleaves AT-I to yield the active pressor octapeptide angiotensin II (AT-II), while concomitantly inactivating the potent vasodilator, bradykinin [3,7]. In addition to the adverse effects of the prolonged use of ACE inhibitors as antihypertensive medication, the alternative ACE-independent, chymase-mediated conversion of AT-I to AT-II in certain organs [8] presents further challenges for the management of hypertension. Therefore, safer antihypertensive agents with the capacity to modulate multiple blood regulation pathways are urgently needed. Given the oft-touted safety of bioactive compounds of biogenic origin in contradistinction to chemically synthesized agents (drugs), various investigators [6,9,10,11,12] have explored the possibility of developing safer but effective antihypertensive agents from animal and plant food proteins in the last few years.

Flaxseed (linseed or *Linum usitatissimum*) which was once typically used only for the production of oil and paint, and later as a fibre-rich source of the heart’s healthy α-linolenic acid (an ω-3 fatty acid) [13], has received significant research attention recently. This is due to the successful investigation of alkali-extracted proteins and enzyme-digested protein hydrolysate samples from its underutilized meal (a by-product of commercial flaxseed oil production) for various salutary benefits including antihypertensive, antidiabetic, antifungal, and antioxidant activities [6,14,15,16]. Additionally, the high quality flaxseed proteins are rich in branched-chain amino acids (BCAA) [17], which have been demonstrated to be potentially important components of antihypertensive peptides [18]. Therefore, the choice of flaxseed as the source of food proteins used in this work was not only to meet the main objective of producing unique thermoase-derived antihypertensive bioactive peptides from flax but would also increase the value added utilization and economic importance of flaxseed meal. The work also investigated the potential role of defined peptide sizes obtained from membrane ultrafiltration as a determinant of peptide antihypertensive activity using spontaneously hypertensive rats (SHR).

## 2. Results and Discussion

### 2.1. Inhibition of in Vitro ACE and Human Recombinant Renin Activities by Flaxseed Protein Hydrolysates (FPH)

Figure 1 shows the differential inhibition of ACE by flaxseed protein hydrolysates (FPH) samples obtained following digestion with various concentrations of thermoase GL-30. The highest inhibitory value of 87% was recorded for the FPH sample obtained at the 3% thermoase concentration and this level of ACE inhibition was significantly (*p* < 0.05) higher than the values obtained for all the other protein hydrolysate samples. While the increases in enzyme concentration from 0.5% to 1%, and from 1% to 1.5% resulted in statistically significant differences in the percentage of ACE inhibition, neither increasing the enzyme concentration from 1.5% to 2%, nor from 2% to 2.5% produced any difference in ACE inhibition of statistical significance. The results suggest that increasing enzyme concentration between 0.5% and 1.5% was important for the production of antihypertensive peptides whereas a similar increase in enzyme concentration between 1.5% and 2% yielded negligible or no differences in ACE-inhibiting peptides.

**Figure 1:** Percentage (mean ± standard error) angiotensin I-converting enzyme- (ACE-) inhibitory activity of flaxseed protein hydrolysates (FPH) digested with thermoase GL-30 (0.5%–3%). Bars with different letters have mean values that are significantly different (*p* < 0.05).

Flaxseed proteins are known to have a high concentration of BCAA [17], which have been shown to be important in the inhibition of ACE activity [18], and thus in potentiating the antihypertensive property of bioactive peptides. Since thermoase GL-30 is an isoform of thermolysin which is known for its specificity in cleaving at the *N*-terminal regions of aromatic, bulky and hydrophobic amino acid residues and thus releasing BCAA (leucine, isoleucine and valine) [18,19], it was carefully chosen to yield a high proportion of BCAA-enriched hydrolysates. Interestingly, the FPH sample at the 3% enzyme concentration which inhibited ACE activity the most has the highest percentage (15.80%) of BCAA as shown in Table 1 which is comparable to the BCAA content of 16.79% obtained by Udenigwe and Aluko [18] after sequential hydrolysis of flaxseed protein isolate (FPI) with thermolysin and pronase. Given the previously reported capacity of hydrophobic amino acids (HAA) for inhibiting ACE activity [9,20], their relatively high content in all the FPH samples suggests important *in vitro* antihypertensive properties and a potential role in the reduction of elevated blood pressure. Percentage ACE-inhibitory activity by the six different FPH samples, which ranged from 79% to 87% is comparable to the percentage ACE-inhibitory activities of about 84% and 82%, respectively, at the same final assay concentration of 1 mg/mL reported for ACE inhibition by thermolysin-digested (pH 8.0, 50 °C, 4 h) rapeseed protein samples [21] and pepsin-digested (pH 3.0, 37 °C, 4 h) canola protein samples [20] using the *N*-(3-[2-furyl]acryloyl)-phenylalanylglycylglycine (FAPGG)-based spectrophotometric method (described in Section 3.2.3.). However, the observed values in this work are significantly (*p* < 0.05) higher than the 70.4% ± 0.4% ACE inhibition obtained using a hippuryl-l-histidyl-l-leucine (HHL)-based chromatographic method, which was reported for thermolysin-digested (pH 8.0, 60 °C, 3 h) rapeseed protein samples [10]. All the FPH samples showed at least 28.0% ± 0.46% renin inhibition (Figure 2) with the percentages of renin-inhibitory activities of 39% and 40% at the 2.5% and 3% enzyme concentrations, respectively, being significantly (*p* < 0.05) higher than the *in vitro* percentage inhibition ranging from 28% to 32% which was observed at the 0.5%–2% enzyme concentrations. The highest renin-inhibitory activity of 40.0% ± 0.94% which was observed with FPH at the 3% enzyme concentration suggests that just as with ACE inhibition, increasing the concentration of thermoase to 3% resulted in a marked increase in renin inhibition, probably because greater amounts of peptides were liberated from the native protein at higher enzyme concentration.

**Figure 2:** Percentage (mean ± standard error) renin-inhibitory activity of flaxseed protein hydrolysates (FPH) after sample hydrolysis with a range (0.5%–3%) of thermoase GL-30 concentrations. Bars with different letters have mean values that are significantly different (*p* < 0.05).

**Table 1:** Percentage amino acid (AA) compositions of flaxseed protein meal (FPM), isolate (FPI), and hydrolysates (FPH) samples digested at different thermoase-GL 30 concentrations (0.5%–3%).

AA	FPM	FPI	0.5% FPH	1.0% FPH	1.5% FPH	2.0% FPH	2.5% FPH	3.0% FPH
ASX	9.76	9.39	11.61	11.53	11.01	11.74	11.59	11.41
THR	3.70	3.24	3.50	3.51	3.44	3.55	3.50	3.37
SER	5.05	4.73	5.21	5.19	5.14	5.29	5.19	4.92
GLX	20.92	23.44	22.18	21.47	22.56	21.91	21.59	21.44
PRO	3.95	3.73	4.49	4.43	4.29	4.50	4.31	4.36
GLY	6.14	6.00	5.47	5.37	5.56	5.41	5.34	5.27
ALA	4.59	4.04	4.52	4.56	4.28	4.57	4.51	4.54
CYS	1.80	2.13	1.35	1.27	1.58	1.34	1.35	1.32
VAL	5.17	4.85	5.02	5.18	4.97	5.07	5.02	5.53
MET	1.70	1.77	1.22	1.20	1.28	1.09	1.17	1.14
ILE	4.15	3.80	4.19	4.35	4.11	4.19	4.16	4.61
LEU	5.97	5.62	5.57	5.71	5.63	5.71	5.64	5.66
TYR	2.29	2.35	2.45	2.52	2.51	2.54	2.50	2.45
PHE	4.73	4.82	5.11	5.21	5.11	5.18	5.10	5.19
HIS	2.45	2.33	2.34	2.40	2.30	2.37	2.36	2.34
LYS	4.18	3.81	3.23	3.17	3.29	3.20	3.21	3.19
ARG	10.63	11.59	11.82	11.91	11.32	11.62	11.98	11.83
TRP	1.40	1.45	1.29	1.31	1.39	1.37	1.38	1.34
AAA	8.42	8.62	8.85	9.03	9.01	9.08	8.97	8.98
BCAA	15.29	14.27	14.79	15.23	14.71	14.97	14.81	15.80
HAA	35.75	34.55	35.22	35.72	35.15	35.55	35.11	36.13

ASX = aspartic acid and asparagine; THR = threonine; SER = serine; GLX = glutamic acid and glutamine; PRO = proline; GLY = glycine; ALA = alanine; CYS = cysteine; VAL = valine; MET = methionine; ILE = isoleucine; LEU = leucine; TYR = tyrosine; PHE = phenylalanine; HIS = histidine; LYS = lysine; ARG = arginine; TRP = tryptophan; AAA = aromatic amino acid; BCAA = branched-chain amino acid; HAA = hydrophobic amino acid.

The afore-stated inhibition values of *in vitro* renin activity at the 2.5% and 3% enzyme concentrations are comparable to the values of about 49% and 40%, respectively, which were reported for renin inhibition at the same final assay concentration of 1 mg/mL by trypsin-digested canola proteins [20] and rapeseed protein sequentially digested by 4% pepsin-pancreatin [21]. However, while >2.5 mg/mL of 1% thermolysin-digested flaxseed proteins was reported to accomplish 50% *in vitro* inhibition of human recombinant renin in a previous study [6], the concentration of 1 mg/mL used in the present study resulted in ≈40% renin inhibitory activity at the 2.5% and 3% enzyme concentrations. Higher renin-inhibitory activity values of about 45%, 52% and 82%, respectively, have been reported for rapeseed protein hydrolysates produced from 4% thermolysin, 4% proteinase K, and 4% alcalase digestion [21]. However, a 4% alcalase protein hydrolysate of African yam bean was reported to have a renin inhibition value of about 38% which is similar to the results for the 2.5% and 3% thermoase enzyme concentrations in the present study [22]. Furthermore, significantly (*p* < 0.05) lower values than those observed for the 2.5% and 3% thermoase concentrations in this study have been reported for 2% alcalase-hydrolysed chicken thigh skin protein (≈16% inhibition), 3% alcalase-hydrolysed chicken breast protein (≈24%) and 4% alcalase hydrolysed chicken breast protein (≈9%) as well as chicken breast skin protein sequentially hydrolysed with 4% pepsin-pancreatin (≈14%) [12]. As was suggested by Udenigwe *et al.* [6], the considerably lower inhibition of renin by enzyme-derived food protein hydrolysates in comparison to their ACE inhibition could be as a result of the presence of more ACE-inhibitory peptides than similar renin inhibitors in enzymatically-digested food proteins thus resulting in a relatively easier inhibition of ACE than renin.

The FPH samples obtained at the 2.5% and 3% enzyme concentrations showed the highest inhibition of ACE and renin and were consequently subjected to membrane fractionation as well as used for *in vivo* systolic blood pressure measurements in spontaneously hypertensive rats.

### 2.2. ACE and Renin Inhibition by FPH Membrane Fractions

FPH samples obtained using 2.5% (2.5% FPH) or 3% (2.5% FPH) thermoase concentration were separated by membrane ultrafiltration and the defined peptide size fractions used for *in vitro* ACE and renin inhibition tests. As shown in Figure 3, membrane ultrafiltration influenced the antihypertensive properties of the <1 kDa FPH fractions at both the 2.5% and 3% enzyme concentrations as evidenced by the considerable increase in ACE inhibition (up to 90%) relative to the inhibition of ACE activity by the unfractionated protein hydrolysate samples (Section 2.1). This level of ACE inhibition by the <1 kDa peptide fraction is the highest recorded both for the unfractionated protein hydrolysate and the membrane fractions, and is significantly (*p* < 0.05) higher than the ACE-inhibitory activity of the 1–3, the 3–5 and the 5–10 kDa fractions. No significant difference was observed in the ACE-inhibitory activity of the <1 kDa peptide fractions obtained from 2.5% FPH (2.5% FPH* < 1 kDa) or 3.0% FPH concentrations (3% FPH* < 1 kDa), which indicates that peptide size at the <1 kDa level played a greater role in ACE inhibition than the amount of enzyme used for proteolysis. For the 3 kDa molecular weight cut-off (MWCO) membrane, peptide fractions from the 3% enzyme-derived hydrolysate (3% FPH* 1–3 kDa) displayed a significantly (*p* < 0.05) higher inhibition of ACE than the corresponding peptide fractions from the 2.5% enzyme hydrolysate (2.5% FPH* 1–3 kDa). As the MWCO increased from 3 to 10 kDa, the ability of the fractions to inhibit ACE activity markedly decreased although the amount of enzyme used for digestion remained the same. While increasing MWCO and the correspondingly larger peptide sizes clearly resulted in a decrease in peptide fraction ACE inhibitory potential, interestingly, there was no significant difference between the 5–10 kDa peptide fraction at the 3% enzyme concentration (3% FPH* 5–10 kDa) and those of 1–3 and 3–5 kDa at the 2.5% enzyme concentration (2.5% FPH* 1–3 kDa and 2.5% FPH* 3–5 kDa, respectively), which indicates a lack of influence at high enzyme concentrations.

The ACE inhibition of 90% shown by the two <1 kDa fractions in Figure 3 is similar to previously reported results of ≈84% and 88%, respectively, for <1 kDa membrane fractions from 4% thermolysin- and 4% proteinase K-digested rapeseed proteins [21], comparable to results obtained with peptide fractions of the same size from chicken thigh skin protein hydrolysate at 3% alcalase [12] concentration (≈82% inhibition) but significantly (*p* < 0.05) higher than the ≈78% inhibition of <1 kDa membrane fractions obtained following the hydrolysis of chicken breast skin protein with 1% pepsin-pancreatin [12]. The 2.5% FPH* 1–3 KDa peptide fractions from the current work inhibited ACE activity to a degree similar to the 86% inhibition reported for peptide fractions of an identical size from 4% thermolysin-hydrolyzed rapeseed proteins but they were significantly (*p* < 0.05) more potent ACE inhibitors than peptide fractions 1–3 kDa in size from both 3% alcalase-digested chicken thigh skin protein hydrolysate (with ACE inhibitory activity of ≈62%) and chicken breast skin protein hydrolysed using 1% pepsin-pancreatin (≈68% inhibition) [12]. Similarly, at inhibition percentages ranging from 86% to 88%, the 3–5 and 5–10 kDa peptide fractions inhibited ACE activity at levels that are comparable to previously reported values of 82%–85% inhibition for 4% thermolysin-digested rapeseed protein hydrolysate fractions of similar sizes [21] but showed significantly higher inhibitory activity than membrane fractions of identical sizes from chicken protein hydrolysate samples [12]. Altogether, the most potent ACE-inhibitory fractions from this study (2.5% FPH* < 1 kDa and 3% FPH* < 1 kDa) showed a degree of inhibition higher than the maximum of 80% inhibition reported for arginine-rich flaxseed cationic fractions at a final assay concentration of 1 mg/mL [23], which may be due to the presence of more hydrophobic and aromatic amino acid residues in the peptide fractions from the current study [24] as shown in Table 1.

**Figure 3:** Percentage (mean ± standard error) of ACE-inhibitory activity of flaxseed protein hydrolysate (FPH) membrane ultrafiltration fractions after hydrolysis of isolated flaxseed proteins with 2.5% or 3.0% thermoase GL-30 and passing the hydrolysates through molecular weight cut-offs (MWCOs) of 1, 3, 5 and 10 kDa. Bars with different letters have mean values that are significantly different (*p* < 0.05).

As Figure 4 shows, renin activity was moderately inhibited by virtually all the membrane fractions. While the renin-inhibitory activities of the 2.5% FPH* 3–5 kDa, 2.5% FPH* 5–10 kDa and 3% FPH* 5–10 kDa fractions ranged from 37% to 38%, the rest of the membrane fractions accomplished at least 40% *in vitro* inhibition of renin activity. The results for membrane fractions that show <40% renin-inhibitory activity are similar to the 36% and 38% inhibition, respectively, reported at the same final assay concentration for the 3–5 kDa fractions from flavourzyme-hydrolyzed rapeseed proteins and 1–3 kDa membrane fractions from alcalase-hydrolyzed chicken thigh skin proteins. Similarly, the >40% renin-inhibitory values are comparable to previous results reported for <1 kDa rapeseed protein hydrolysates and 3–5 kDa chicken thigh skin protein hydrolysates [12,21]. Although no significant difference was observed in the inhibition of renin activity between the <1 and 1–3 kDa fractions at the two different enzyme concentrations used, at 40% renin inhibitory activity, the 3% FPH* 3–5 kDa fraction significantly (*p* < 0.05) inhibited renin activity more than the 38% inhibition observed with the 2.5% FPH* 3–5 kDa fractions. This difference could be attributed to the release of a greater amount of peptides from the native protein structure at the higher enzyme concentration. The results generally suggest higher renin inhibitory activity by the smaller peptides than those larger in size—a trend which has been reported in previous studies [9,21].

**Figure 4:** Percentage (mean ± standard error) renin-inhibitory activity of flaxseed protein hydrolysate (FPH) membrane ultrafiltration fractions after hydrolysis of isolated flaxseed proteins with 2.5% or 3.0% thermoase GL-30 and passing the hydrolysates through MWCOs of 1, 3, 5 and 10 kDa. Bars with different letters have mean values that are significantly different (*p* < 0.05).

Inhibition of renin activity by the 2.5% FPH* < 1 kDa and 3% FPH* < 1 kDa fractions is similar to the 39% and 40% inhibition, respectively, which were previously reported for membrane fractions that contain an identical peptide size obtained from chicken thigh skin proteins digested with 3% alcalase [12] and rapeseed proteins digested with 4% alcalase [21]. The 2.5% FPH* 1–3 kDa and 3% FPH* 1–3 kDa fractions also inhibited renin activity to a degree similar to the 39% renin inhibitory activity accomplished by peptide membrane fractions of an identical size from rapeseed proteins sequentially digested with 4% pepsin and pancreatin [21]. However, the 49% and 57% reported inhibition of renin activity by 1–3 kDa membrane fractions from 4% alcalase- and 4% proteinase K-digested rapeseed proteins respectively are considerably higher than the inhibitory activity shown by fractions of identical size (2.5% FPH* 1–3 kDa and 3% FPH* 1–3 kDa) from the current study [12]. Inhibition of renin activity by the 2.5% FPH* 3–5 kDa and 3% FPH* 3–5 kDa fractions are comparable to the 38% and 42% inhibition respectively reported for fractions of corresponding size obtained from 4% flavourzyme and 4% alcalase hydrolysates of rapeseed [21]. However, the renin-inhibitory activity of 2.5% FPH* 5–10 kDa and 3% FPH* 5–10 kDa fractions was each considerably higher than the 24%, 26% and 23% inhibition respectively accomplished by peptide fractions of the same size from 4% alcalase, 4% pepsin-pancreatin and 4% flavourzyme hydrolysate fractions of rapeseed proteins but substantially lower than the inhibition of 55% and 57% correspondingly shown by 4% proteinase K- and 4% thermolysin-digested rapeseed protein hydrolysate fractions of the same size [21]. A previous work that screened cationic membrane fractions from flaxseed proteins sequentially digested with trypsin and pronase reported a maximum renin inhibition of 44.5% at a peptide final assay concentration of 0.75 mg/mL. In the current work, although the FPH peptide fractions were used at a slightly higher final assay concentration of 1 mg/mL in a similarly-designed assay, renin-inhibitory values akin to that of the previous work were obtained [23]; the differences may be attributed to variations in the type of amino acid residues present in both fractions [23].

### 2.3. In Vivo Antihypertensive Activity of FPH and FPH Membrane Fractions

As illustrated in Figure 5, Figure 6 and Figure 7, all the FPH and membrane fraction samples administered to the spontaneously hypertensive rats (SHR) significantly (*p* < 0.05) lowered systolic blood pressure (SBP) at all measured time points better than phosphate buffered saline (PBS), thus providing *prima facie* evidence and preliminary confirmation that the test samples do indeed possess *in vivo* antihypertensive effects. The protein hydrolysate which showed the highest SBP reduction (−29 mm Hg after 4 h) was the 3% FPH sample while the unhydrolyzed flaxseed protein isolate (FPI) had the least BP-lowering activity (−4 to −5 mm Hg after 4–6 h) as shown in Figure 5. The SBP-lowering activities of the 2.5% FPH and 3% FPH samples after 2–8 h were comparable to that of captopril (used as a positive control and at a dosage 20 times lower), thus suggesting the potential of the peptide samples to rapidly lower blood pressure on a short term basis. However, the blood pressure-lowering ability of captopril was significantly (*p* < 0.05) better than those of the protein hydrolysates after 24 h of oral administration. Although the hypotensive effect of FPI slightly increased from −2 mm Hg after 2 h to ≈−4 to −5 mm Hg after 4–6 h, the two FPH samples showed significantly (*p* < 0.05) higher SBP decreases than the FPI sample at every time point. The results support the fundamental principle that protein hydrolysates contain more rapidly absorbable peptides than the unhydrolysed protein isolate. Additionally, since proteolysis of native proteins must take place before absorption of any antihypertensive peptides, it is logical to expect weak FPI antihypertensive effect on a short-term basis when compared to FPH samples that contain predigested peptides.

The SBP-lowering activity of the two hydrolysate samples were similar but had diminished considerably after 24 h post-oral administration with a maximum value of −13 mmHg, which is still significantly (*p* < 0.05) higher than the maximum effect (−5 mmHg after 6 h) of the unhydrolysed protein (FPI).

In Figure 6 and Figure 7, the 2.5% FPH and 3% FPH samples both showed significantly (*p* < 0.05) larger decreases in SBP than some of the corresponding membrane permeates (3–5 and 5–10 kDa) after 2 and 4 h. However, at both the 6 and 8 h marks, the SBP-reducing effect of some of the membrane permeates (1–3 and 3–5 kDa) was significantly (*p* < 0.05) greater than that of their corresponding protein hydrolysates. This could be as a result of the fact that the membrane fractions had longer intrinsic synergistic effects or less antagonistic effects due to the higher level of peptide homogeneity when compared to the high peptide heterogeneity in the unfractionated protein hydrolysates. Therefore, the protein hydrolysates may be useful ingredients to formulate fast-acting antihypertensive products while the membrane fractions would be suitable for extended-release type of antihypertensive formulations.

**Figure 5:** Effects of 2.5% and 3% enzymatic flaxseed protein hydrolysate (FPH), and flaxseed protein isolate (FPI) samples on systolic blood pressure (SBP) of spontaneously hypertensive rats (SHR) after oral gavage. Rats were administered with FPH and FPI using a dose of 200 mg protein/kg rat body weight (BW) while the positive control, captopril was given at 10 mg/kg body weight. Saline was used as negative control. Bars with different letters have mean SBP values that are significantly (*p* < 0.05) different.

**Figure 6:** Effects of 2.5% enzymatic flaxseed protein hydrolysate (FPH), membrane ultrafiltration peptide fractions and flaxseed protein isolate (FPI) on systolic blood pressure (SBP) of spontaneously hypertensive rats (SHR) after oral gavage. Rats were administered with FPH, FPH fractions and FPI using a dose of 200 mg protein/kg rat body weight (BW) while the positive control, captopril was given at 10 mg/kg body weight. Saline was used as the negative control. Bars with different letters have mean SBP values that are significantly (*p* < 0.05) different.

Among the peptide fractions from the 2.5% FPH sample (Figure 6), the hypotensive activities of 2.5% FPH* < 1 kDa and 2.5% FPH* 1–3 kDa tended to be the highest after 2 h indicating their possible ability to lower blood pressure on a short term basis but also suggesting that the larger peptides in the 5 and 10 kDa fractions might not have been as efficiently absorbed as the smaller <1 and 1–3 kDa peptides in such a short amount of time. Alternatively, it is possible that the longer peptides undergo initial hydrolysis to release active fragments that are then subsequently absorbed; this will delay the antihypertensive effect. The significant (*p* < 0.05) increases in the BP-reducing effect of the larger peptides (3–5 and 5–10 kDa) after 4 and 6 h lends credence to this reasoning. Remarkably, all the membrane fractions from both protein hydrolysate samples maintained significant hypotensive effects after 24 h (approximately −8 mm Hg in the least).

**Figure 7:** Effects of 3% enzymatic flaxseed protein hydrolysate (FPH), membrane ultrafiltration peptide fractions and flaxseed protein isolate (FPI) samples on systolic blood pressure (SBP) of spontaneously hypertensive rats (SHR) after oral gavage. Rats were administered with FPH, FPH fractions and FPI using a dose of 200 mg protein/kg rat body weight (BW) while the positive control, captopril was given at 10 mg/kg body weight. Saline was used as a blank. Bars with different letters have mean SBP values that are significantly (*p* < 0.05) different.

Contrary to what was observed with the 2.5% FPH fractions, the 3–5 and 5–10 kDa fractions of the 3.5% FPH sample (Figure 7) were very effective in lowering elevated blood pressure in SHR. In fact, unlike in the fractions from the 2.5% FPH sample where 2.5% FPH* 1–3 kDa was responsible for the largest decrease in blood pressure (−34 mm Hg) after 6 h, 3% FPH* 3–5 kDa exerted the highest blood pressure-lowering effect of −37 mm Hg after 8 h among the fractions from the 3% FPH sample. This difference could be as a result of, among other things, the difference in the concentration of peptides liberated by the different enzyme concentrations and additional processing of the peptides in the gastrointestinal tract of the SHR.

Similar results have been obtained with the enzymatic hydrolysate samples of hemp seed protein hydrolysate [9] (after 2 h in comparison to 2.5% FPH at the same time point) and pepsin-digested canola protein hydrolysate after 8 h [20] (compared to 3% FPH after the same number of hours). Although a reduction in SBP of about −15 mm Hg, which is comparable to that of 2.5% FPH after 8 h, was reported with an oral dose of sweet potato protein hydrolysate [25] lower than the 200 mg/kg BW used in this study at the same hour mark, the SBP-lowering effects of the flaxseed protein hydrolysate and membrane fractions used in this study lasted longer (an average of −12 mm Hg after 24 h) when compared to that of the enzyme-digested sweet potato proteins (nearly zero after 24 h).

## 3. Experimental Section

### 3.1. Materials

Captopril, cellulase (from *Aspergillus niger*; approximately 0.8 units/mg protein), *N*-(3-[2-furyl]acryloyl)-phenylalanylglycylglycine (FAPGG), and ACE (from rabbit lung, ≥2.0 units/mg protein) were procured from Sigma-Aldrich (St. Louis, MO, USA). Thermoase GL-30 was from Amano Enzyme Inc. (Nagoya, Japan), while a human recombinant Renin Inhibitor Screening Assay Kit was purchased from Cayman Chemicals (Ann Arbor, MI, USA). Pulverized, defatted flaxseed meal was obtained from Bioriginal Foods and Science Corporation (Saskatoon, SK, Canada) while SHR were supplied by Charles River Laboratories (Montreal, PQ, Canada). The ultrafiltration membranes of 1, 3, 5 and 10 kDa MWCO and other analytical grade reagents were procured from Fischer Scientific (Oakville, ON, Canada).

### 3.2. Methods

#### 3.2.1. Preparation of Flaxseed Protein Isolate (FPI)

The protein components of defatted flaxseed flour were isolated using an improved modification [6] of the alkali extraction/acid precipitation method [26]. Defatted flaxseed flour (5%, *w*/*v*, dry weight basis) was suspended in ultrapure, deionized water and continuously stirred using a magnetic stirrer until a uniformly dispersed but highly viscous slurry was obtained. The suspension was heated to 37 °C and adjusted to pH 5.0 using 0.5 M HCl. Thereafter, cellulase (1%, *w*/*w*; activity of powder, 1.44 U/mg) was added to the slurry to initiate fibre hydrolysis. After 4 h of reaction, the suspension was cooled to 4 °C and adjusted to pH 10.0 with the addition of 0.5 M NaOH for the alkaline extraction step. The alkaline suspension was mixed for 1 h at room temperature, which was followed by centrifugation at 15,000× *g* for 30 min; the supernatant was collected and adjusted to pH 4.2 by the gradual step-wise addition of 0.5 M HCl. The supernatant obtained after a second round of centrifugation was then discarded while the precipitated protein curd was washed thrice with acidified distilled water (pH 4.2) before being suspended in a small volume of deionized water. The suspension was subsequently adjusted to pH 7.0 before it was freeze-dried as the FPI.

#### 3.2.2. Hydrolysis of Isolated Flaxseed Proteins and Production of Membrane Fractions

After suspending the FPI in deionized water (5%, *w*/*v*, protein basis), the suspension was stirred with a magnetic stirrer, heated to 37 °C and adjusted to pH 8.0 before the addition of thermoase GL-30. Following addition of enzyme to the slurry at the appropriate enzyme-substrate ratio *E*/*S* (0.5%–3%), the reaction mixture was heated to 37 °C, adjusted to pH 8.0 using 2 M NaOH and stirred for 4 h [6]; temperature and pH were maintained constant during the reaction period. The reaction was terminated when the enzyme was inactivated by immersing the reaction vessel in a boiling water bath for 15 min while the precipitation of undigested proteins was achieved first by using 1 M HCl to adjust the mixture to pH 4.0 followed by centrifugation for 30 min at 15,000× *g*. The supernatant which contains the peptides of interest was then sequentially passed through ultrafiltration membranes beginning with the MWCO of 1 kDa, and continuing (using the retentate) through those of the 3 kDa, 5 kDa (retentate from 3 kDa) and 10 kDa (retentate from 5 kDa) to obtain permeates with, peptides sizes of <1, 1–3, 3–5 and 5–10 kDa, respectively. The permeates were then freeze-dried and stored at −20 °C until used for subsequent tests. The percentage protein content of the FPI, FPH and membrane fractions was determined by a modified Lowry’s method using bovine serum albumin as standard [27].

#### 3.2.3. ACE-Inhibitory Activity of FPH and Membrane Fractions

The FPH and membrane fractions were assayed for inhibitory activity against ACE as previously described [6,28]. Briefly, 1 mL of 0.5 mM FAPGG (dissolved in 50 mM Tris–HCl buffer containing 0.3 M NaCl, pH 7.5) was combined with 20 µL ACE (1 U/mL; final activity of 20 mU), and 200 µL of 50 mM Tris–HCl containing 6.1 mg/mL of the appropriate sample (FPH or membrane fraction) for a final peptide concentration of 1 mg/mL. The decreased absorbance at 345 nm, due to ACE-catalyzed cleavage of the Phe-Gly peptide bond of FAPGG, was recorded at regular intervals for 2 min at room temperature using a Varian Cary 50-UV/Visible spectrophotometer (Varian, Victoria, Australia). Tris–HCl buffer was used instead of peptide samples in the blank experiment. All experiments were performed in triplicate. ACE activity was expressed as rate of disappearance of FAPGG (Δ*A*/min) and inhibitory activity was calculated as follows:

Percentage ACE inhibition = 1 − [Δ*A*·min^−1^_(sample)_/Δ*A*·min^−1^_(blank)_] × 100 (1)

where Δ*A*·min^−1^_(sample)_ and Δ*A*·min^−1^_(blank)_ are the reaction rates in the presence and absence of FPH or membrane fractions respectively.

#### 3.2.4. Renin-Inhibitory Activity of FPH and Membrane Fractions

The ability of the FPH and membrane fractions to inhibit the activity of human recombinant renin *in vitro* was determined by fluorescence spectrometry using the Renin Inhibitor Screening Assay Kit according to a previously described method [6]. The total assay volume of 190 µL included 19 µL of 10 mg/mL FPH or membrane fraction which had earlier been dissolved in 50 mM Tris–HCl buffer containing 100 mM NaCl (pH 8.0), 10 µM Arg-Glu(EDANS)-Ile-His-Pro-Phe-His-Leu-Val-Ile-His-Thr-Lys(Dabcyl)-Arg (renin substrate dissolved in dimethyl sulphoxide), and human recombinant renin. Tris–HCl buffer was used instead of the flaxseed peptide solution in the blank experiment while each sample well contained a final peptide concentration of 1 mg/mL. The 96-well plate containing the various thoroughly mixed reaction mixtures was pre-warmed to 37 °C for 15 min to attain thermal equilibrium before monitoring the periodic increases in fluorescence intensity using a fluorometric microplate reader (Spectra MAX Gemini, Molecular Devices, Sunnyvale, CA, USA) with excitation and emission wavelengths set at 340 and 490 nm, respectively. The percentage inhibition was calculated as follows:

Renin inhibition (%) = [(FIU·min^−1^_(blank)_ − FIU·min^−1^_(sample)_/FIU·min^−1^_(blank)_] × 100 (2)

where FIU·min^−1^_(blank)_ and FIU·min^−1^_(sample)_ are the fluorescent intensity in the absence and presence of peptides, respectively.

#### 3.2.5. Amino Acid Composition Analysis

The amino acid profiles of FPH samples were determined using an HPLC Pico-Tag method following the digestion of samples with 6 M HCl [29]. The cysteine and methionine contents were determined after oxidation with performic acid [30] while the samples were analyzed for tryptophan content following alkaline hydrolysis [31].

#### 3.2.6. Evaluation of FPH and Membrane Fractions for Antihypertensive Activity in Spontaneously Hypertensive Rats (SHR)

All animal experiments were conducted according to protocol F011-015/1/2, which was approved by the University of Manitoba Animal Protocol and Management Review Committee, as prescribed by the guidelines of the Canadian Council on Animal Care Ethics. Male SHR (20-week-old; 250–300 g body weight, BW) with tail SBP of over 150 mmHg were kept at the Animal Care Facility of the Richardson Centre for Functional Foods and Nutraceuticals, University of Manitoba. Rats were housed individually using steel cages in a room maintained under a 12 h light-dark cycle, temperature of 23 °C (±2 °C) and relative humidity of 50%. The SHR were fed a standard chow diet and tap water *ad libitum* before and after oral gavage. FPI (from Section 3.2.1), 2.5% FPH and 3.0% FPH samples obtained by the digestion of FPI with 2.5% and 3.0% thermoase GL-30, respectively, the membrane fractions (<1, 1–3, 3–5 and 5–10 kDa in size) from the ultrafiltration of each of the two FPH samples, as well as captopril were each dissolved in phosphate-buffered saline (PBS), pH 7.2. The samples (each at 200 mg/kg BW), PBS (used as negative control), and captopril (10 mg/kg BW; used as positive control) were administered to the SHR by oral gavage followed by measurement of systolic blood pressure (SBP) by tail-cuff plethysmography (Mouse Rat Tail Cuff Blood Pressure System, IITC Life Science, Woodland Hills, CA, USA) at 2, 4, 6, 8 and 24 h in rats mildly anesthetized for 4 min with 4% isoflurane [9,32]. The gas flow chamber, maintained at 37 °C, was designed to include positive pressure ventilation in order to sustain independent ventilatory function and attenuate isoflurane-induced depression of spontaneous ventilation in the animals. The entire procedure was optimized to ensure that the SHR regained consciousness within 3–4 min of being taken out of the chamber, thus giving enough time for the measurement of blood pressure while the animals were still chemically restrained, and ensuring negligible or no depression of SBP by the inhalational anesthetic agent. Baseline (time zero) SBP was measured before the administration of samples, and the change in SBP (ΔSBP, mm Hg) was calculated by subtracting the data for the different time points from their respective baseline data.

#### 3.2.7. Statistical Analysis

All assays were conducted in replicates of three and data are reported as mean ± standard deviation. Values were tested for statistical significance of difference using Duncan’s multiple range test (*p* < 0.05) with the Statistical Analysis Systems, SAS, software version 9.2 (SAS, Cary, NC, USA).

## 4. Conclusions

The digestion of isolated flaxseed proteins using various concentrations of thermoase yielded SBP-lowering peptides with great potential for use in the formulation of antihypertensive nutraceuticals. The *in vivo* and *in vitro* hypotensive effects of the samples were influenced by the concentration of enzyme used for protein hydrolysis as well as the peptide size. Although the samples showed very high ACE-inhibitory activity, their inhibition of renin activity was only moderate. Nevertheless, both the unfractionated hydrolysate and the peptide fractions significantly (*p* < 0.05) lowered SBP in SHR from 2–24 h after oral administration, highlighting their potential to provide fast relief from elevated blood pressure on a short term basis. Furthermore, the strong SBP-reducing effect of the unfractionated hydrolysate samples also suggests that while membrane purification may increase their potency (as seen with the 2.5% FPH* 1–3 kDa and 3% FPH* 3–5 kDa fractions), subjecting them to further purification could be avoided as a cost-saving measure during formulation of functional foods and nutraceuticals. Overall, the 3% FPH would be preferred as the best blood pressure-reducing agent among all the samples, simply because of the higher potency when compared to 2.5% FPH; the higher potency could enable lower dosage and hence lower cost of the 3% FPH.
